# Topical Tacrolimus and Periodontal Therapy in the Management of a Case of Oral Chronic GVHD Characterized by Specific Gingival Localization

**DOI:** 10.1155/2014/127219

**Published:** 2014-01-02

**Authors:** Davide Conrotto, Roberto Broccoletti, Paola Carcieri, Luisa Giaccone, Paolo G. Arduino

**Affiliations:** ^1^Department of Surgical Sciences, Oral Medicine Section, CIR Dental School, University of Turin, Via Nizza 230, 10126 Turin, Italy; ^2^Division of Haematology, Azienda Ospedaliera Città della Salute e della Scienza, University of Turin, Corso Bramante 88, 10126 Turin, Italy

## Abstract

*Background*. Chronic graft versus host disease (cGVHD) is a complication following bone marrow transplantation. The oral lesions are difficult to control with a systemic pharmacological therapy. *Case Description*. A 63-year-old female patient, who underwent an allogeniec transplantation for acute myeloid leukemia, developed a chronic oral and cutaneous GVHD. The patient was treated with topical tacrolimus 0.1%, twice daily for two months, and underwent a protocol of oral hygiene characterized by 3 appointments of scaling, root planning, and daily oral hygiene instructions. The patient showed marked resolution of gingival lesions and a significant improvement of related pain and gingival inflammatory indexes. *Clinical Implications*. This case report suggests that treatment with topical tacrolimus and professional oral hygiene may be helpful in the management of chronic oral GVHD with severe gingival involvement.

## 1. Introduction

Chronic graft versus host disease (cGVHD) is a complication following bone marrow transplantation, which frequently involves the oral mucosa [1]. When affected, oral tissues present with lichenoid-like lesions, erythema, and ulcerations; lesions on gingiva can induce a “desquamative gingivitis,” similar to that of oral lichen planus and mucous membrane pemphigoid, presenting with epithelial desquamation, erythematous zones, and erosive lesions on the gingival tissue. Patients usually complain of pain and difficulty in eating, speaking in and swallowing, with a significant decrease in the quality of life. Oral hygiene is particularly difficult and the periodontal status often worsens [2].

Tacrolimus is a macrolide immunosuppressant derived from *Streptomyces tsukubaensis*. It is a relatively selective inhibitor of calcineurin and it was initially developed as a systemic agent to lessen allograft rejection [3, 4].

Previous reports suggest that topical therapy with tacrolimus can be helpful in the management of oral lesions caused by GVHD [5–7]. In some of those patients, however, the response on gingival lesions is often partial. We report a case in which the combined treatment of topical tacrolimus and periodontal therapy allowed satisfactory control of the severe gingival profile due to oral cGVHD.

## 2. Case Presentation

A 63-year-old female patient, who underwent an allogeneic transplantation for acute myeloid leukemia about 5 years ago, with a complete clinical remission, presented with chronic, biopsy proven, oral, and cutaneous GVDH of moderate degree. The patient was referred to the Unit of Oral Medicine Section of the University of Turin (Italy), complaining of extreme gingival pain. Oral manifestations were characterized by atrophic and erosive lichenoid-like lesions on buccal and gingival mucosa. Even if an immunosuppressive therapy with systemic cyclosporine (Sandimmun Neoral, Novartis Farma S.p.A., Origgio, Varese, Italy) and systemic prednisone (Deltacortene, Bruno Farmaceutici S.p.A., Roma, Italy) was carried out, the management of the oral disease was unsuccessful. The patient complained of severe intraoral symptoms, which made chewing, speaking, and oral hygiene procedures very difficult.

Patient was informed about the experimental protocol and signed a consent form. The ethics review board of the Lingotto Dental School approved the study. She received a comprehensive periodontal examination at baseline visit, including full mouth plaque scores (FMPS) and full mouth bleeding on probing scores (FMBS). We started the treatment with tacrolimus ointment (Protopic 0.1% ointment, Astellas Pharma S.p.A, Carugate, Milano, Italy) twice daily for two months. Patient was carefully instructed on how to apply the medications: finger rub application on dried lesions after meals without eating, drinking, or speaking for at least half an hour afterwards. Antimycotic treatment was also added, consisting of miconazole gel (Daktarin 2% oral gel, Janssen-Cilag S.p.A., Cologno Monzese, Milano, Italy) applied once daily plus 0.12% chlorhexidine mouth rinse without alcohol (Curasept A.D.S. 0.12%, Curaden Healthcare S.r.l., Saronno, Varese, Italy) three times daily. In order to evaluate possible systemic absorption, blood tacrolimus levels were monitored at the beginning and at the end of the two-month protocol. After 2 weeks from the beginning of therapy, she also received a nonsurgical periodontal protocol, including oral hygiene instructions and supra- and subgingival scaling as required. Oral hygiene instructions were given by an experienced dental hygienist, who also provided thorough supragingival scaling and polishing with removal of all deposits and staining, once a week, for three weeks [8]. Patient-related outcomes included pain perception assessed at each visit by Visual Analogue Scale (VAS). The VAS consisted of a 10 cm horizontal line marked with 0 (= no pain) to 10 (= most severe pain experienced). At each visit, the patient was examined by means of record chart compilation, oral examination, registration of symptoms and clinical sings, and periodontal index.

The patient, at the end of the protocol, showed marked resolution of gingival lesions and a significant improvement of buccal lesions (Figure 1). No increase of tacrolimus plasma levels was noticed during the treatment period. A reduction in FMBS, FMPS, and VAS scores was observed (data not shown). No reported complications or therapy side effects were observed.

## 3. Discussion

The pathogenesis of plaque-related periodontal disease involves local activation of the immune system induced by bacterial factors [9]. cGVHD is an immunomediated disease [1]; we can postulate that some influences could exist and that a bacterial induced inflammation could amplify the effects of cGVHD on gingival mucosa. Furthermore, dental plaque may aggravate burning sensation and reported symptoms. Despite its limitations, our data proposes that treatment with topical tacrolimus, combined with nonsurgical periodontal therapy and oral hygiene instructions, may be successful in reducing clinical gingival inflammation and improving patient-related outcomes in a case of cGVHD with severe gingival involvement. We postulate that the topical drug is useful in creating a preliminary breakdown in inflammation and so allowing an efficient nonsurgical periodontal therapy consisting of scaling and effective bacterial plaque control, which can later represent an essential approach for the control of gingival lesions and permit competent oral hygiene. Topical tacrolimus is safe for short periods, but the systemic absorption should, however, be monitored [10].

To the best of our knowledge, this is the first case ever reported of a patient with gingival cGVHD treated with nonsurgical periodontal therapy combined with topical tacrolimus. Previously, topical tacrolimus has been successfully used for the treatment of oral cGVHD alone [6, 11, 12] or in combination with systemic steroid [7] or photopheresis [13]. The gingival involvement was detailed by Sánchez and coworkers [5], who reported a successful treatment with topical tacrolimus three times daily.

The importance of a careful plaque removal and the maintenance of periodontal health are unequivocal for many chronic diseases that can induce a desquamative gingivitis, as oral lichen planus or pemphigoid [8]. Probably something similar can happen for cGVHD too.

Systemic calcineurin inhibitors have been shown to have oncogenic properties mainly linked to the production of cytokines that promote tumour growth, metastasis, and angiogenesis. To date there is no strong evidence that topical application of calcineurin inhibitors may be associated with an increased risk of tumours [4]. However, the benefits of tacrolimus should be weighed against its potential risks, and diligent long-term follow-up should be carried out by well-trained oral clinicians.

The positive clinical results obtained with a standard professional oral hygiene and nonsurgical periodontal protocol could serve as a basis for recommending this as a first line therapeutic intervention, especially in patients with pure gingival involvement, in order to decrease gingival inflammation and related pain and help affected patients in maintaining a good oral hygiene. Studies on large groups of patients are, however, suggested.

## Figures and Tables

**Figure 1:** Sixty-three-year-old female patient with gingival and buccal cGVHD at baseline ((a), (b)), and after the proposed protocol ((c), (d)).
